# Bayesian and Non-Bayesian Reliability Estimation of Stress-Strength Model for Power-Modified Lindley Distribution

**DOI:** 10.1155/2022/1154705

**Published:** 2022-02-22

**Authors:** Abdulhakim A. Al-Babtain, I. Elbatal, Ehab M. Almetwally

**Affiliations:** ^1^Department of Statistics and Operations Research, King Saud University, Riyadh 11362, Saudi Arabia; ^2^Department of Mathematics and Statistics-College of Science, Imam Mohammad Ibn Saud Islamic University, Riyadh, Saudi Arabia; ^3^Department of Statistics, Faculty of Business Administration, Delta University of Science and Technology, Gamasa, Egypt; ^4^Faculty of Graduate Studies for Statistical Research, Cairo University, Giza 12613, Egypt

## Abstract

A two-parameter continuous distribution, namely, power-modified Lindley (PML), is proposed. Various structural properties of the new distribution, including moments, moment-generating function, conditional moments, mean deviations, mean residual lifetime, and mean past lifetime, are provided. The reliability of a system is discussed when the strength of the system and the stress imposed on it are independent. Maximum-likelihood estimation of the parameters and their estimated asymptotic standard errors are derived. Bayesian estimation methods of the parameters with independent gamma prior are discussed based on symmetric and asymmetric loss functions. We proposed using the MCMC technique with the Metropolis–Hastings algorithm to approximate the posteriors of the stress-strength parameters for Bayesian calculations. The confidence interval for likelihood and the Bayesian estimation method is obtained for the parameter of the model and stress-strength reliability. We prove empirically the importance and flexibility of the new distribution in modeling with real data applications.

## 1. Introduction

Modeling and evaluating lifespan data are critical in many practical fields, including medical, engineering, and finance, to name a few. To model such data, a variety of lifetime distributions, such as the exponential, Weibull, gamma, and Rayleigh distributions, for example, and their generalizations, have been used (see, e.g., Gupta and Kundu [1] and Nadarajah and Kotz [2]). Because of the form of the failure rate function, which can be monotonically declining, increasing, or constant in behavior, as well as nonmonotone, bathtub-shaped, or even unimodal, each distribution has its unique peculiarities.

The Lindley distribution was introduced by Lindley [3] as a new distribution useful to analyze lifetime data, especially in applications modeling stress-strength reliability, earthquakes, floods, engineering, physics, quality control, and medicine as well as for modeling lifetime data. Ghitany et al. [4] investigated the Lindley distribution's properties using a rigorous mathematical approach. They also demonstrated that the Lindley distribution models' waiting periods and survival times are better than the exponential distribution in a numerical example. Mazucheli and Achcar [5] investigated the Lindley distribution's applications to competing hazard lifetime data. The Lindley distribution also has some useful qualities for lifetime data analysis, including closed forms for the survival and hazard functions and strong fit flexibility.

The cumulative distribution function (cdf) and probability density function (pdf) of Lindley distribution are given by

(1) $$\begin{array}{c} F\left(x,\theta \right)=1-e^{-\theta x}\left[1+\frac{\theta x}{\theta +1}\right],x>0,\theta >0, \end{array}$$

(2) $$\begin{array}{c} f\left(x,\theta \right)=\frac{\theta^{2}}{\theta +1}\left(1+x\right)e^{-\theta x};x>0,\theta >0. \end{array}$$

Recently, Chesneau et al. [6] have introduced a general family of Lindley, called modified Lindley (ML) distribution based on the use of a new tuning function, which aims at modulating the polynomial term in the definition of the cdf given by (1). The cdf and pdf of the ML distribution are given by

(3) $$\begin{array}{c} G\left(x;\theta \right)=1-e^{-\theta x}\left[1+\frac{\theta x}{\theta +1}e^{-\theta x}\right],x>0, \end{array}$$

(4) $$\begin{array}{c} g\left(x;\theta \right)=\frac{\theta }{\theta +1}e^{-2\theta x}\left[\left(1+\theta \right)e^{\theta x}+2x\theta -1\right]. \end{array}$$

Using power transformation of a random variable may offer a more flexible distribution model by adding a new parameter. Mazucheli et al. [7] proposed the power Lindley (PL) as a new extension of the Lindley distribution based on (1) and by using the transformation *X*=*T*^1/*β*^. This model provides more flexibility than the Lindley distribution in terms of the shape of the density and hazard rate functions as well as its skewness and kurtosis. The cdf and pdf of the PL distribution are given by

(5) $$\begin{array}{c} G\left(x,\theta ,\beta \right)=1-e^{-\theta x^{\beta }}\left[1+\frac{\theta x^{\beta }}{\theta +1}\right], \end{array}$$

(6) $$\begin{array}{c} g\left(x,\theta ,\beta \right)=\frac{\theta^{2}\beta }{\theta +1}x^{\beta -1}e^{-\theta x^{\beta }}\left(1+x^{\beta }\right), \end{array}$$

respectively, where *θ*  > 0 is a scale parameter and *β*  > 0 is a shape parameter. In this present work, an attempt to propose a new flexible distribution by the transformation technique. The proposed distribution is called the power-modified Lindley (PML). The rationality of considering the PML distribution is that it equips the most famous extensions of the ML.

In statistics, inferring stress-strength reliability is an important issue of study. It has a wide range of practical applications. *R* = *P*(*Y* < *X*) is a measure of component reliability in stress-strength modeling. When *X* equals *Y*, the component fails or malfunctions, where *X* is subject to *Y*. In electrical and electronic systems, *R* might also be considered. The estimation of the stress-strength reliability *R*=*P*(*Y* < *X*), where *X* and *Y* follow the power-modified Lindley distribution, is the topic of this study.

The power-modified Lindley distribution's derivation is largely focused with its usage in data analysis, making it valuable in a variety of fields, particularly those involving lifespan analysis. This model has not been investigated before, as far as we know, despite the fact that we feel it plays a significant role in reliability analysis. The likelihood estimator (LE) is obtained. An asymptotic confidence interval is created using the asymptotic distribution. The Bayesian estimator of stress-strength *R* and its accompanying credible interval are obtained using the Gibbs sampling technique. Finally, we discuss the flexibility of the proposed model for three different applications of real data.

The rest of the article is organized as follows. In Section 2, we introduce a new distribution. In Section 3,we provide some basic statistical properties of this distribution, including moment, moment-generating function, incomplete moments, and mean deviations. In Section 4, Bayesian and likelihood methods of parameters are derived. In Section 5, the reliability parameter related to the stress-strength model is derived. In Section 6, we use the different methods of confidence intervals for model parameters. Some simulations to investigate the accuracy and reliability of the maximum likelihood estimators are performed in Section 7. Three applications to real datasets prove empirically the flexibility of the new model introduced in Section 7. Finally, Section 9 offers some concluding remarks.

## 2. Power-Modified Lindley Distribution

A new extension of the modified Lindley distribution is proposed by considering the power transformation *X*=*T*^1/*α*^. The distribution of *X* is referred to as power-modified Lindley (PML) distribution. The cdf of the PML is defined by

(7) $$\begin{array}{c} F\left(x,\theta ,\alpha \right)=1-e^{-\theta x^{\alpha }}\left[1+\frac{\theta x^{\alpha }}{\theta +1}e^{-\theta x^{\alpha }}\right],x>0. \end{array}$$

The corresponding pdf and hazard rate function are, respectively, given by

(8) $$\begin{array}{c} f\left(x,\theta ,\alpha \right)=\frac{\theta \alpha }{\theta +1}e^{-2\theta x^{\alpha }}x^{\alpha -1}\left[\left(1+\theta \right)e^{\theta x^{\alpha }}+2\theta x^{\alpha }-1\right], \end{array}$$

(9) $$\begin{array}{c} h\left(x,\theta ,\alpha \right)=\frac{\theta \alpha x^{\alpha -1}\left[\left(1+\theta \right)e^{\theta x^{\alpha }}+2\theta x^{\alpha }-1\right]}{\left(\theta +1\right)e^{\theta x^{\alpha }}\left[1+\theta x^{\alpha }/\theta +1e^{-\theta x^{\alpha }}\right]}, \end{array}$$

where *θ* > 0 is a scale parameter and *α*  > 0 is a shape parameter. Hereafter, a random variable *X* that has the pdf given in (8) is denoted by *X*∽PML(*θ*, *α*).

Figure 1 explains how the behavior of pdf and hazard rate of PML distribution is affected for shapes by increasing the value of parameters *α* and *θ*.

## 3. Statistical Properties

Moments, moment-generating function, conditional moments, mean deviation, and moments of residual and reversed residual lifetimes are some of the essential statistical properties of the MPL distribution presented in this section.

### 3.1. Moments and Associated Measures

Moments can be used to investigate some of the most essential properties and characteristics of a distribution. The *r*^th^ moment of *X* denoted as *μ*_*r*_′ can be obtained from (8) as follows:

(10) $$\begin{array}{c} \mu_{r}^{\prime }=\int_{0}^{\infty }x^{r}f\left(x\right)\text{dx}\\ =\int_{0}^{\infty }\frac{\theta \alpha }{1+\theta }e^{-2\theta x^{\alpha }}x^{r+\alpha -1}\left[\left(1+\theta \right)e^{\theta x^{\alpha }}+2\theta x^{\alpha }-1\right]\text{dx}\\ =\frac{\left(1+\theta \right)\Gamma \left(r/\alpha +1\right)}{\alpha \theta^{r/\alpha +1}}+\frac{\Gamma \left(r/\alpha +2\right)}{\alpha {\left(2\theta \right)}^{r/\alpha +1}}-\frac{\Gamma \left(r/\alpha +1\right)}{\alpha {\left(2\theta \right)}^{r/\alpha +1}}\\ =\frac{\Gamma \left(r/\alpha +1\right)}{\theta^{r/\alpha }}\left[1+\frac{r/\alpha }{2^{r/\alpha +1}\left(1+\theta \right)}\right]. \end{array}$$

Set *r*=1, and we have *E*(*X*)=*μ*_1_′=Γ(1/*α*+1)/*θ*^1/*α*^[1+1/*α*/2^1/*α*1^(1+*θ*)]. The *n*_*th*_ central moment of *X* is given by

(11) $$\begin{array}{c} M_{n}=E{\left(X-\mu_{1}^{\prime }\right)}^{n}\\ =\overset{\infty }{\underset{r=0}{\sum }}\left(\begin{array}{c} n\\ r \end{array}\right){\left(-\mu_{1}^{\prime }\right)}^{n-r}\mu_{r}^{\prime }. \end{array}$$

Also, the skewness and kurtosis coefficients of *X* are, respectively, defined by *S*_*k*_=*μ*_3_′ − 3*μ*_2_′*μ*+2*μ*^3^/[*μ*_2_′ − *μ*^2^]3/2 and *k*_*u*_=*μ*_4_′ − 4*μ*_3_′*μ*+6*μ*_2_′*μ*^2^ − 3*μ*^4^/[*μ*_2_′ − *μ*^2^]^2^. The moment-generating function *M*_*X*_(*t*) given by (8) can be obtained as follows:

(12) $$\begin{array}{c} M_{X}\left(t\right)=E\left(e^{tx}\right)\\ =\overset{\infty }{\underset{r=0}{\sum }}\frac{t^{r}}{r!}\mu_{r}^{\prime }\left(x\right)\\ =\overset{\infty }{\underset{r=0}{\sum }}\frac{t^{r}}{r!}\frac{\Gamma \left(r/\alpha +1\right)}{\theta^{r/\alpha }}\left[1+\frac{r/\alpha }{2^{r/\alpha +1}\left(1+\theta \right)}\right]. \end{array}$$

### 3.2. Conditional Moments

The incomplete moments, the mean residual lifetime function, and the mean inactivity time function are also useful properties for lifetime models. The Bonferroni and Lorenz curves are the most common applications of the first incomplete moment. In economics, dependability, demographics, insurance, and medical, these curves are extremely valuable. It is useful to know the *s*_th_ lower and upper incomplete moments of *X* in lifetime models, which are defined by *ϑ*_*s*_(*t*)=*E*(*X*^*s*^∣*X* > *t*)=∫_*t*_^*∞*^*x*^*s*^*f*(*x*)dx and *ψ*_*s*_(*t*)=*E*(*X*^*s*^∣*X* < *t*)=∫_0_^*t*^*x*^*s*^*f*(*x*)dx, respectively; for any real *s* > 0, the *s*_th_ upper incomplete moment of PML distribution is

(13) $$\begin{array}{c} \vartheta_{s}\left(t\right)=\int_{t}^{\infty }x^{s}f\left(x\right)\text{dx}=\\ =\int_{0}^{\infty }\frac{\theta \alpha }{1+\theta }e^{-2\theta x^{\alpha }}x^{r+\alpha -1}\left[\left(1+\theta \right)e^{\theta x^{\alpha }}+2\theta x^{\alpha }-1\right]\text{dx}\\ =\frac{1}{\theta^{s/\alpha }}\left\{\Gamma \left(\frac{s}{\alpha }+1,\theta t^{\alpha }\right)+\frac{1}{\left(\theta +1\right)2^{s/\alpha +1}}\left[\Gamma \left(\frac{s}{\alpha }+2,2\theta t^{\alpha }\right)-\Gamma \left(\frac{s}{\alpha }+1,2\theta t^{\alpha }\right)\right]\right\}, \end{array}$$

where Γ(*s*, *t*)=∫_*t*_^*∞*^*x*^*s*−1^*e*^−*x*^dx denotes the upper incomplete gamma function. The first incomplete moment of *X*, marked by, *ϑ*_1_(*t*), is computed using (15) by setting *s*=1 as

(14) $$\begin{array}{c} \vartheta_{1}\left(t\right)=\frac{1}{\theta^{1/\alpha }}\left\{\Gamma \left(\frac{1}{\alpha }+1,\theta t^{\alpha }\right)+\frac{1}{\left(\theta +1\right)2^{1/\alpha +1}}\left[\Gamma \left(\frac{1}{\alpha }+2,2\theta t^{\alpha }\right)-\Gamma \left(\frac{1}{\alpha }+1,2\theta t^{\alpha }\right)\right]\right\}. \end{array}$$

Similarly, the *s*_th_ lower incomplete moment of PML distribution is

(15) $$\begin{array}{c} \psi_{s}\left(t\right)=\int_{0}^{t}x^{s}f\left(x\right)\text{dx}\\ =\frac{1}{\theta^{s/\alpha }}\left\{\xi \left(\frac{s}{\alpha }+1,\theta t^{\alpha }\right)+\frac{1}{\left(\theta +1\right)2^{s/\alpha +1}}\right.\left.\left[\xi \left(\frac{s}{\alpha }+2,2\theta t^{\alpha }\right)-\xi \left(\frac{s}{\alpha }+1,2\theta t^{\alpha }\right)\right]\right\}, \end{array}$$

where *ξ*(*s*, *t*)=∫_0_^*t*^*x*^*s*−1^*e*^−*x*^dx is the lower incomplete gamma function. The first incomplete moment of *X*, denoted by, *ψ*_1_(*t*), is computed using (15) by setting *s*=1 as

(16) $$\begin{array}{c} \psi_{1}\left(t\right)=\frac{1}{\theta^{1/\alpha }}\left\{\xi \left(\frac{1}{\alpha }+1,\theta t^{\alpha }\right)+\frac{1}{\left(\theta +1\right)2^{1/\alpha +1}}\left[\xi \left(\frac{1}{\alpha }+2,2\theta t^{\alpha }\right)-\xi \left(\frac{1}{\alpha }+1,2\theta t^{\alpha }\right)\right]\right\}. \end{array}$$

The mean residual lifetime (MRL) function (or the life expectancy at age *t*) represents the expected additional life length for a unit, which is alive at age *t*. The MRL of PML distribution is given by

(17) $$\begin{array}{c} m_{X}\left(t\right)=E\left(X|X>t\right)\\ =\frac{\vartheta_{1}\left(t\right)}{\bar{F}\left(t\right)}-t\\ =\frac{1}{\bar{F}\left(t\right)\theta^{1/\alpha }}\left\{\Gamma \left(\frac{1}{\alpha }+1,\theta t^{\alpha }\right)+\frac{1}{\left(\theta +1\right)2^{1/\alpha +1}}\left[\Gamma \left(\frac{1}{\alpha }+2,2\theta t^{\alpha }\right)-\Gamma \left(\frac{1}{\alpha }+1,2\theta t^{\alpha }\right)\right]\right\}-t. \end{array}$$

Also, the mean inactivity time (MIT) represents the waiting time elapsed since the failure of an item on condition that this failure had occurred in (0; *t*). The MIT of *X* is defined (for *t* > 0) by

(18) $$\begin{array}{c} \tau_{X}\left(t\right)=E\left(X|X<t\right)\\ =t-\frac{\psi_{1}\left(t\right)}{F\left(t\right)}\\ =t-\frac{\theta^{1/\alpha }}{F\left(t\right)}\left\{\xi \left(\frac{1}{\alpha }+1,\theta t^{\alpha }\right)+\frac{1}{\left(\theta +1\right)2^{1/\alpha +1}}\left[\xi \left(\frac{1}{\alpha }+2,2\theta t^{\alpha }\right)-\xi \left(\frac{1}{\alpha }+1,2\theta t^{\alpha }\right)\right]\right\}. \end{array}$$

Another application of the conditional moments is the mean deviation about the mean (*μ*) and about the median (*M*). For the PML distribution, the mean deviation about the mean and mean deviation about the median, respectively, given by

(19) $$\begin{array}{c} \zeta_{\mu }\left(x\right)=\int_{0}^{\infty }|x-\mu |f\left(x\right)\text{dx}\\ =2\mu F\left(\mu \right)-2\mu +2\vartheta_{1}\left(\mu \right). \end{array}$$

(20) $$\begin{array}{c} \zeta_{M}\left(x\right)=\int_{0}^{\infty }|x-M|f\left(x\right)\text{dx}\\ =2\vartheta_{1}\left(M\right)-\mu , \end{array}$$

where *ϑ*_1_(*μ*) and *ϑ*_1_(*M*) can be determined from equation (13). In addition, *F*(*μ*) can be computed from equation (7).

The Bonferroni and Lorenz curves were proposed now. Bonferroni [8] and the Gini indices have applications in domains other than economics, such as reliability, demography, insurance, and medicine. The Bonferroni curve is given by

(21) $$\begin{array}{c} B\left(p\right)=\frac{1}{p\mu }\int_{0}^{q}xf\left(x\right)\text{dx}\\ =\frac{1}{p\mu \theta^{1/\alpha }}\left\{\xi \left(\frac{1}{\alpha }+1,\theta q^{\alpha }\right)+\frac{1}{\left(\theta +1\right)2^{1/\alpha +1}}\left[\xi \left(\frac{1}{\alpha }+2,2\theta q^{\alpha }\right)-\xi \left(\frac{1}{\alpha }+1,2\theta q^{\alpha }\right)\right]\right\}, \end{array}$$

where *μ*=*E*(*X*) and *q*=*F*^−1^(*p*). Also, Lorenz curve is given by

(22) $$\begin{array}{c} L\left(p\right)=\frac{1}{\mu }\int_{0}^{q}xf\left(x\right)\text{dx}\\ =\frac{1}{\mu \theta^{1/\alpha }}\left\{\xi \left(\frac{1}{\alpha }+1,\theta q^{\alpha }\right)+\frac{1}{\left(\theta +1\right)2^{1/\alpha +1}}\left[\xi \left(\frac{1}{\alpha }+2,2\theta q^{\alpha }\right)-\xi \left(\frac{1}{\alpha }+1,2\theta q^{\alpha }\right)\right]\right\}. \end{array}$$

### 3.3. Moments of Residual and Reversed Residual Lifetimes

The mean residual lifetime and mean past lifetime have very important to describe the different maintenance strategies. The *n*_th_-order moment of the residual life is obtained by the following formula:

(23) $$\begin{array}{c} \mu_{n}\left(t\right)\\ =E\left[{\left(X-t\right)}^{n}|X>t\right]\\ =\frac{1}{\bar{F}\left(t\right)}\int_{t}^{\infty }{\left(x-t\right)}^{n}f\left(x\right)\text{dx},n\geq 1\\ =\frac{1}{\bar{F}\left(t\right)}\overset{n}{\underset{s=0}{\sum }}{\left(-t\right)}^{n-s}\left(\begin{array}{c} n\\ s \end{array}\right)\int_{t}^{\infty }x^{s}f\left(x\right)\text{dx}\\ =\frac{1}{\bar{F}\left(t\right)}\overset{n}{\underset{s=0}{\sum }}{\left(-t\right)}^{n-s}\left(\begin{array}{c} n\\ s \end{array}\right)\vartheta_{s}\left(t\right). \end{array}$$

Setting *s*=1, we get the MRL. On the other hand, the *n*_th_ moment of the reversed residual life (inactivity time) is given by

(24) $$\begin{array}{c} m_{s}\left(t\right)=E\left({\left(t-X\right)}^{n}|X\leq t\right)\\ =\frac{1}{F\left(t\right)}\int_{0}^{t}{\left(t-x\right)}^{n}f\left(x\right)\text{dx},n\geq 1\\ =\frac{1}{F\left(t\right)}\overset{n}{\underset{s=0}{\sum }}{\left(-t\right)}^{n-s}\left(\begin{array}{c} n\\ s \end{array}\right)\int_{t}^{\infty }x^{s}f\left(x\right)\text{dx}\\ =\frac{1}{\bar{F}\left(t\right)}\overset{n}{\underset{s=0}{\sum }}{\left(-t\right)}^{n-s}\left(\begin{array}{c} n\\ s \end{array}\right)\psi_{s}\left(t\right), \end{array}$$

where the mean past lifetime can be obtained using (15) by setting *s*=1.

## 4. Bayesian and Non-Bayesian Estimation

In this section, the estimation procedures by Bayesian and non-Bayesian estimation methods of the parameters *α* and *θ* of the PML distribution are obtained. We provided non-Bayesian estimation for the PML model as maximum likelihood (ML) and Bayesian estimation by using different loss functions such as square error loss function (SELF), the LINEX loss function, and the entropy loss function.

### 4.1. Likelihood Estimation Method

Let *X*_1_, *X*_2_,…, *X*_*n*_ be a random sample of size *n* from PML distribution with parameters *θ* and *α*. The likelihood function for the vector of parameters *ϕ*=(*θ*, *α*) can be written as

(25) $$\begin{array}{c} L\left(\phi \right)=\alpha^{n}{\left(\frac{\theta }{\theta +1}\right)}^{n}e^{-2\theta \sum_{i=1}^{n}x_{i}^{\alpha }}\prod_{i=1}^{n}x_{i}^{\alpha -1}\left[\left(1+\theta \right)e^{\theta x_{i}^{\alpha }}+2\theta x_{i}^{\alpha }-1\right]. \end{array}$$

The log-likelihood function for the vector of parameters *ϕ* can be written as

(26) $$\begin{array}{c} \log\;L=n\text{log}\theta +n\;\log\;\alpha -n\;\log\left(1+\theta \right)-2\theta \overset{n}{\underset{i=1}{\sum }}x_{i}^{\alpha }+\overset{n}{\underset{i=1}{\sum }}\log\left[\left(1+\theta \right)e^{\theta x_{i}^{\alpha }}+2\theta x_{i}^{\alpha }-1\right]. \end{array}$$

The maximum-likelihood estimate for *θ* and *α* is obtained by solving the nonlinear equations obtained by differentiating (26) with respect to *θ* and *α*. The score vector components, say *U*_*n*_(*ϕ*)=∂*L*/∂*ϕ*=[∂*L*/∂*θ*, ∂*L*/∂*α*]^*T*^, are given by

(27) $$\begin{array}{c} \frac{\partial \;\log\;L}{\partial \theta }=\frac{n}{\theta }-\frac{n}{\left(1+\theta \right)}-2\overset{n}{\underset{i=1}{\sum }}x_{i}^{\alpha }+\overset{n}{\underset{i=1}{\sum }}\frac{e^{\theta x_{i}^{\alpha }}\left(1+x_{i}^{\alpha }+\theta x_{i}^{\alpha }\right)+2x_{i}^{\alpha }}{\left(1+\theta \right)e^{\theta x_{i}^{\alpha }}+2\theta x_{i}^{\alpha }-1}. \end{array}$$

(28) $$\begin{array}{c} \frac{\partial \;\log\;L}{\partial \alpha }=\frac{n}{\alpha }-2\theta \overset{n}{\underset{i=1}{\sum }}x_{i}^{\alpha }\log\;x_{i}+\overset{n}{\underset{i=1}{\sum }}\frac{\theta \left(1+\theta \right)e^{\theta x_{i}^{\alpha }}x_{i}^{\alpha }\log\;x_{i}+2\theta x_{i}^{\alpha }\log\;x_{i}}{\left(1+\theta \right)e^{\theta x_{i}^{\alpha }}+2\theta x_{i}^{\alpha }-1}. \end{array}$$

By solving the nonlinear system *U*_*n*_(*ϕ*)=0, the maximum LE (MLE) of *ϕ*, say $\hat{\phi }$, is obtained. These equations cannot be solved analytically; however, they can be solved numerically using statistical software using iterative approaches. To get the estimate $\hat{\phi }$, we can utilize iterative techniques like a Newton–Raphson algorithm.

### 4.2. Prior Distribution

We assume that the parameters *α* and *θ* are independently distributed according to the gamma distribution for building Bayesian estimation. Let *α* and *θ* have gamma priors with scale and shape parameters *q*_*j*_ and *w*_*j*_, respectively. A proportionate representation of the joint prior density of *α* and *θ* is the following:

(29) $$\begin{array}{c} \mathbb{C}\left(\alpha ,\theta \right)\propto \theta^{w_{2}-1}\alpha^{w_{1}-1}\exp\left\{-\left(\theta q_{2}+\alpha q_{1}\right)\right\},\theta ,\alpha >0,q_{j},w_{j}>0;j=1,2. \end{array}$$

### 4.3. Hyperparameter Elicitation

The informative priors will be used to elicit the hyperparameters. The mean and variance using the maximum-likelihood estimates of PML distribution *α* and *θ* will be equated with the mean and variance of the considered priors (gamma priors) *α*^*j*^ and *θ*^*j*^, where *j*=1,……, *k* and *k* is the number of samples available from the PML distribution. We can derive the mean and variance of alpha and theta by equating them with the mean and variance of gamma priors. We get

(30) $$\begin{array}{c} \frac{1}{k}\overset{k}{\underset{j=1}{\sum }}\alpha^{j}=\frac{w_{1}}{q_{1}},\\ \frac{1}{k-1}\overset{k}{\underset{j=1}{\sum }}{\left(\alpha^{j}-\frac{1}{k}\overset{k}{\underset{j=1}{\sum }}\alpha^{j}\right)}^{2}=\frac{w_{1}}{q_{1}^{2}}. \end{array}$$

(31) $$\begin{array}{c} \frac{1}{k}\overset{k}{\underset{j=1}{\sum }}\theta^{j}=\frac{w_{2}}{q_{2}},\\ \frac{1}{k-1}\overset{k}{\underset{j=1}{\sum }}{\left(\theta^{j}-\frac{1}{k}\overset{k}{\underset{j=1}{\sum }}\theta^{j}\right)}^{2}=\frac{w_{2}}{q_{2}^{2}}. \end{array}$$

The estimated hyperparameters can now be stated as follows after solving the preceding two equations:

(32) $$\begin{array}{c} w_{1}=\frac{{\left(1/k\sum_{j=1}^{k}\alpha^{j}\right)}^{2}}{1/k-1\sum_{j=1}^{k}{\left(\alpha^{j}-1/k\sum_{j=1}^{k}\alpha^{j}\right)}^{2}},\\ q_{1}=\frac{1/k\sum_{j=1}^{k}\alpha^{j}}{1/k-1\sum_{j=1}^{k}{\left(\alpha^{j}-1/k\sum_{j=1}^{k}\alpha^{j}\right)}^{2}}. \end{array}$$

(33) $$\begin{array}{c} w_{2}=\frac{{\left(1/k\sum_{j=1}^{k}\theta^{j}\right)}^{2}}{1/k-1\sum_{j=1}^{k}{\left(\theta^{j}-1/k\sum_{j=1}^{k}\theta^{j}\right)}^{2}},\\ q_{2}=\frac{1/k\sum_{j=1}^{k}\theta^{j}}{1/k-1\sum_{j=1}^{k}{\left(\theta^{j}-1/k\sum_{j=1}^{k}\theta^{j}\right)}^{2}}. \end{array}$$

### 4.4. Posterior Distribution

The joint posterior distribution can be expressed as the product of likelihood function equation (25) and the joint prior function (29). Then, the joint posterior density function of *ϕ* is

(34) $$\begin{array}{c} G\left(\phi |x\right)=A\alpha^{n+w_{1}-1}\theta^{n+w_{2}-1}{\left(\frac{1}{\theta +1}\right)}^{n}e^{-\theta \left(q_{2}+2\sum_{i=1}^{n}x_{i}^{\alpha }\right)}e^{-\alpha \left(\sum_{i=1}^{n}\text{ln}\left(x_{i}\right)+q_{1}\right)}\prod_{i=1}^{n}\left[\left(1+\theta \right)e^{\theta x_{i}^{\alpha }}+2\theta x_{i}^{\alpha }-1\right]. \end{array}$$

In actuality, the posterior density's normalization constant *𝔸* is often intractable, requiring an integral over the parameter space.

### 4.5. Symmetric Loss Function

The symmetric loss function is the squared-error loss function (SELF), which is defined by

(35) $$\begin{array}{c} L_{S}\left(\tilde{\Omega },\Omega \right)\propto {\left(\tilde{\Omega }-\Omega \right)}^{2}, \end{array}$$

Then, the Bayesian estimator of Ω under SELF is the average:

(36) $$\begin{array}{c} {\tilde{\Omega }}^{S}=E_{\Omega }\left(\Omega \right). \end{array}$$

### 4.6. Asymmetric Loss Function

In this section, we discussed the LINEX and entropy loss function, which are the most famous loss functions.

#### 4.6.1. LINEX Loss Function

Varian and Savage [9] presented a highly useful asymmetric loss function, which has lately been employed in different works [10, 11] and [12]. This function is known as the LINEX loss function, according to linear exponentially. The LINEX loss function can be stated as follows, assuming that the minimal loss occurs at $\tilde{\Omega }=\Omega$:

(37) $$\begin{array}{c} L_{L}\left(\tilde{\Omega },\Omega \right)\propto e^{c\left({\tilde{\Omega }}^{L}-\Omega \right)}-c\left({\tilde{\Omega }}^{L}-\Omega \right)-1;c\neq 0, \end{array}$$

where $\tilde{\Omega }$ is any estimate of the parameter Ω and *c* is the shape parameter. The value of *c* determines the shape of this loss function. Then, the Bayes estimator of Ω under entropy loss function is

(38) $$\begin{array}{c} {\tilde{\Omega }}^{L}=\frac{-1}{c}\ln\left[E_{\Omega }\left(e^{-c\Omega }\right)\right]. \end{array}$$

After studying the LINEX loss function, and from Figure 2 which displays LINEX loss with different values of *c*, we note that the function is fairly asymmetric for *c*=1, with $\left({\tilde{\Omega }}^{L}-\Omega \right)>0$, and the function is asymmetric for *c*=−1, with $\left({\tilde{\Omega }}^{L}-\Omega \right)<0$.

#### 4.6.2. Entropy Loss Function

In many practical cases, it appears that expressing the loss in terms of the ratio $\tilde{\Omega }/\Omega$ is more realistic. James and Stein initially proposed the entropy loss function by ratio for estimating the variance-covariance (i.e., dispersion) matrix of the multivariate normal distribution. The entropy loss function is a good asymmetric loss function, according to Calabria and Pulcini [13]. The entropy loss function of the form is considered as follows:

(39) $$\begin{array}{c} L_{E}\left(\tilde{\Omega },\Omega \right)\propto {\left(\frac{\tilde{\Omega }}{\Omega }\right)}^{b}-b\text{ln}\left(\frac{\tilde{\Omega }}{\Omega }\right)-1, \end{array}$$

whose minimum occurs at $\tilde{\Omega }=\Omega$. Then, the Bayes estimator of Ω under entropy loss function is

(40) $$\begin{array}{c} {\tilde{\Omega }}_{E}={\left[E_{\Omega }\left(\Omega^{-b}\right)\right]}^{-1/b}. \end{array}$$

Many authors discussed Bayesian estimation under entropy loss function as Dey et al. They [14] used this loss function for the simultaneous estimation of scale parameters and their reciprocals. Singh et al. [15] used this loss function for Bayesian estimation of the exponentiated gamma parameter.

Figure 3 shows that the Bayesian estimate for the entropy loss function is the same as the Bayesian estimate for the weighted squared-error loss function $\tilde{\Omega }-\Omega /\Omega$ when *b*=1. The Bayesian estimate under the entropy loss function with *b*=−1 and the Bayesian estimate under the squared-error loss function are identical. A positive error $\left(\tilde{\Omega }>\Omega \right)$ has more serious repercussions than a negative error when *b* > 0 and vice versa when *b* < 0. When both $\tilde{\Omega }$ and Ω are measured in a logarithmic scale, the function is virtually symmetric for small |*b*| values, (see Calabria and Pulcini [13] and Schabe [16]):

(41) $$\begin{array}{c} L_{E}\left(\tilde{\Omega },\Omega \right)\propto \frac{b^{2}}{2}{\left(\text{ln}\left(\tilde{\Omega }\right)-\text{ln}\left(\Omega \right)\right)}^{2}. \end{array}$$

### 4.7. Markov Chain Monte Carlo

The MCMC approach will be utilized because these integrals are difficult to solve analytically. Gibbs sampling and more generic Metropolis-within-Gibbs samplers are two prominent subclasses of MCMC algorithms. Gibbs sampling and more generic Metropolis-within-Gibbs samplers are key subclasses of MCMC algorithms. This algorithm was first introduced by Metropolis et al. [17]. For more information, see Soliman et al. [18], Okasha et al. [19], Han [20], Singh et al. [21], and Haj Ahmad et al. [22]. The Metropolis–Hastings (MH) algorithm [23] is similar to acceptance-rejection sampling in that it considers a candidate value derived from a proposal distribution as normal for each iteration of the process [24]. The MH algorithm uses two steps to compute a suitable transition starting at *ϕ*_*i*_=*ϕ*:

1. Draw *ϕ*^*∗*^ from a proposal density as normal distribution as *q*(*ϕ*^*∗*^*|ϕ*).
2. Either retain the current sample *ϕ*_*i*+1_=*ϕ* or transition to *ϕ*_*i*+1_=*ϕ*^*∗*^ with acceptance probability:

(42) $$\begin{array}{c} a_{\phi^{*}|\phi }=\min\left[1,\frac{G\left(\phi^{*}|x\right)q\left(\phi \right)}{G\left(\phi |x\right)q\left(\phi^{*}|\phi \right)}\right]. \end{array}$$

This well-defined transition density not only ensures that the target density remains invariant, but also that the chain converges to its unique invariant density starting from any initial condition under the right conditions *ϕ*.

## 5. Stress-Strength Reliability Computations

In this section, we investigate the reliability parameter related to the *PML* distribution. Let *X* is the strength of a system and *Y* is the stress acting on it has aroused wide concern. If *X* follows PML(*α*, *θ*_1_) and *Y* follows PML(*α*, *θ*_2_) provided *X* and *Y* are the independent random variables. Then, reliability *R*=*P*(*Y* < *X*). Many engineering concepts, such as structures, rocket motor deterioration, static fatigue of ceramic components, fatigue failure of aircraft structures, and the aging of concrete pressure vessel reliability, all benefit from it:

(43) $$\begin{array}{c} R=P\left(Y<X=x\right)\\ =\int_{0}^{\infty }F_{2}\left(x\right)f_{1}\left(x\right)\text{dx}\\ =1-\int_{0}^{\infty }e^{-\theta_{2}x^{\alpha }}\left[1+\frac{\theta_{2}x^{\alpha }}{\theta_{2}+1}e^{-\theta_{2}x^{\alpha }}\right]\frac{\theta_{1}\alpha }{\theta_{1}+1}e^{-2\theta_{1}x^{\alpha }}x^{\alpha -1}\left[\left(1+\theta_{1}\right)e^{\theta_{1}x^{\alpha }}+2\theta_{1}x^{\alpha }-1\right]\text{dx.} \end{array}$$

Setting *t*=*x*^*α*^, we get

(44) $$\begin{array}{c} R=1-\frac{\theta_{1}}{\theta_{1}+1}\int_{0}^{\infty }e^{-\left(2\theta_{1}+\theta_{2}\right)t}\left[\left(1+\theta_{1}\right)e^{\theta_{1}t}+2\theta_{1}t-1\right]\text{d}t-\frac{\theta_{1}\theta_{2}}{\left(\theta_{1}+1\right)\left(\theta_{2}+1\right)}\int_{0}^{\infty }e^{-2\left(\theta_{1}+\theta_{2}\right)t}\left[\left(1+\theta_{1}\right)e^{\theta_{1}t}+2\theta_{1}t-1\right]\text{d}t\\ =1-\frac{\theta_{1}}{\theta_{1}+1}\left[\frac{\theta_{1}+1}{\theta_{1}+\theta_{2}}+\frac{2\theta_{1}}{{\left(2\theta_{1}+\theta_{2}\right)}^{2}}-\frac{1}{2\theta_{1}+\theta_{2}}\right]-\frac{\theta_{1}\theta_{2}}{\left(\theta_{1}+1\right)\left(\theta_{2}+1\right)}\left[\frac{\theta_{1}+1}{\theta_{1}+2\theta_{2}}+\frac{\theta_{1}}{2{\left(\theta_{1}+\theta_{2}\right)}^{2}}-\frac{1}{2\left(\theta_{1}+\theta_{2}\right)}\right]. \end{array}$$

The reliability stress-strength model of PML is shown in Figure 4 with different values of *θ*_1_, and *θ*_2_.

Many authors have recently used likelihood and Bayesian estimation approaches to estimate *R*=*P*(*Y* < *X*=*x*) for various life testing schemes based on various distributions [25–31].

In MLE of the stress-strength model, let *x*_1_, *x*_2_,…, *x*_*n*_ and *y*_1_, *y*_2_,…, *y*_*m*_ be random samples from PML with *α*, *θ*_1_, and *α*, *θ*_2_, respectively. The likelihood function of the stress-strength model for PML distribution can be expressed as

(45) $$\begin{array}{c} L\left(\Phi \right)=\alpha^{n+m}{\left(\frac{\theta_{1}}{\theta_{1}+1}\right)}^{n}{\left(\frac{\theta_{2}}{\theta_{2}+1}\right)}^{m}e^{-2\theta_{1}\sum_{i=1}^{n}x_{i}^{\alpha }-2\theta_{2}\sum_{i=1}^{m}y_{i}^{\alpha }}\prod_{i=1}^{n}x_{i}^{\alpha -1}\left[\left(1+\theta_{1}\right)e^{\theta_{1}x_{i}^{\alpha }}+2\theta_{1}x_{i}^{\alpha }-1\right]\prod_{i=1}^{m}y_{i}^{\alpha -1}\left[\left(1+\theta_{2}\right)e^{\theta_{2}y_{i}^{\alpha }}+2\theta_{2}y_{i}^{\alpha }-1\right], \end{array}$$

where Φ is the vector of parameter as (*α*, *θ*_1_, *θ*_2_). The log-likelihood function of stress-strength model of PML distribution for the vector of parameters *ϕ* can be written as

(46) $$\begin{array}{c} \log\;L\left(\Phi \right)=n\;\log\;\theta_{1}+\left(n+m\right)\log\left(\alpha \right)-n\;\log\left(1+\theta_{1}\right)-m\;\log\left(1+\theta_{2}\right)-2\theta_{1}\overset{n}{\underset{i=1}{\sum }}x_{i}^{\alpha }-2\theta_{2}\overset{m}{\underset{i=1}{\sum }}y_{i}^{\alpha }+\overset{n}{\underset{i=1}{\sum }}\log\left[\left(1+\theta_{1}\right)e^{\theta_{1}x_{i}^{\alpha }}+2\theta_{1}x_{i}^{\alpha }-1\right]+\overset{m}{\underset{i=1}{\sum }}\log\left[\left(1+\theta_{2}\right)e^{\theta_{2}y_{i}^{\alpha }}+2\theta_{2}y_{i}^{\alpha }-1\right]. \end{array}$$

The maximum-likelihood estimate for *θ*_1_, *θ*_2_, and *α* is obtained by solving the nonlinear equations obtained by differentiating (46) with respect to *θ*_1_, *θ*_2_, and *α*. The score vector components, say *U*_*N*_(Φ)=∂log *L*/∂Φ=[∂  log *L*/∂*θ*_1_, ∂log *L*/∂*θ*_2_, ∂log *L*/∂*α*]^*T*^, are given by

(47) $$\begin{array}{c} \frac{\partial \;\log L}{\partial \theta_{1}}=\frac{n}{\theta_{1}}-\frac{n}{\left(1+\theta_{1}\right)}-2\overset{n}{\underset{i=1}{\sum }}x_{i}^{\alpha }+\overset{n}{\underset{i=1}{\sum }}\frac{e^{\theta_{1}x_{i}^{\alpha }}\left(1+x_{i}^{\alpha }+\theta_{1}x_{i}^{\alpha }\right)+2x_{i}^{\alpha }}{\left(1+\theta_{1}\right)e^{\theta_{1}x_{i}^{\alpha }}+2\theta_{1}x_{i}^{\alpha }-1}, \end{array}$$

(48) $$\begin{array}{c} \frac{\partial \;\log L}{\partial \alpha }=\frac{n+m}{\alpha }-2\theta_{1}\overset{n}{\underset{i=1}{\sum }}x_{i}^{\alpha }\log\;x_{i}-2\theta_{2}\overset{m}{\underset{i=1}{\sum }}y_{i}^{\alpha }\log\;y_{i}+\overset{n}{\underset{i=1}{\sum }}\frac{\theta \left(1+\theta_{1}\right)e^{\theta_{1}x_{i}^{\alpha }}x_{i}^{\alpha }\log\;x_{i}+2\theta_{1}x_{i}^{\alpha }\log\;x_{i}}{\left(1+\theta_{1}\right)e^{\theta_{1}x_{i}^{\alpha }}+2\theta_{1}x_{i}^{\alpha }-1}+\overset{m}{\underset{i=1}{\sum }}\frac{\theta_{2}\left(1+\theta_{2}\right)e^{\theta_{2}y_{i}^{\alpha }}y_{i}^{\alpha }\log\;y_{i}+2\theta_{2}y_{i}^{\alpha }\log\;y_{i}}{\left(1+\theta_{2}\right)e^{\theta_{2}y_{i}^{\alpha }}+2\theta_{2}y_{i}^{\alpha }-1}. \end{array}$$

## 6. Confidence Interval

In this section, the asymptotic confidence interval for the MLE method, and credible confidence interval for the Bayesian estimation method has been obtained.

### 6.1. Asymptotic Confidence Interval

The Fisher information matrix (FIM) of a three-dimensional vector Φ=(*α*, *θ*_1_, *θ*_2_) looks like this:

(49) $$\begin{array}{c} I\left(\alpha ,\theta_{1},\theta_{2}\right)=-\left(\begin{array}{ccc} E\left(\frac{\partial^{2}\log\;L}{\partial \alpha^{2}}\right), & E\left(\frac{\partial^{2}\log\;L}{\partial \alpha \;\partial \theta_{1}}\right), & E\left(\frac{\partial^{2}\log\;L}{\partial \alpha \;\partial \theta_{2}}\right),\\ E\left(\frac{\partial^{2}\log\;L}{\partial \theta_{1}\partial \alpha }\right), & E\left(\frac{\partial^{2}\log\;L}{\partial \theta_{1}^{2}}\right), & 0,\\ E\left(\frac{\partial^{2}\log\;L}{\partial \theta_{2}\partial \alpha }\right), & 0, & E\left(\frac{\partial^{2}\log\;L}{\partial \theta_{2}^{2}}\right). \end{array}\right) \end{array}$$

Assume that $\hat{\Phi }$ represents the MLE of Φ. Then, as *n*⟶*∞*, and *m*⟶*∞*,

(50) $$\begin{array}{c} \sqrt{n}\left(\hat{\Phi }-\Phi \right)\overset{D}{⟶}N\left(0,I^{-1}\right). \end{array}$$

The inverse matrix of the FIM *I* is *I*^−1^. This is where we define

(51) $$\begin{array}{c} B=\left(0,\frac{\partial R}{\partial \theta_{1}},\frac{\partial R}{\partial \theta_{2}}\right). \end{array}$$

Then, using the delta approach (for further information, see Ferguson [32]), the asymptotic distribution of $\hat{R}$ is shown to be as follows:

(52) $$\begin{array}{c} \sqrt{n}\left(\hat{R}-R\right)\overset{D}{⟶}N\left(0,\sigma_{R}^{2}\right), \end{array}$$

where *σ*_*R*_^2^=*B*^*T*^*I*^−1^*B* is the asymptotic variance of $\hat{R}$. The approximate 100(1 − *γ*)% confidence interval for *R* can be expressed as $\left(\hat{R}-z_{\gamma /2}{\hat{\sigma }}_{R},\hat{R}+z_{\gamma /2}{\hat{\sigma }}_{R}\right)$, where *z*_*γ*/2_ is the upper *γ*/2 percentile of the standard normal distribution.

### 6.2. Credible Confidence Interval

The highest posterior density (HPD) confidence intervals are used to discuss credible confidence intervals of parameters of this model for the results of the MCMC. The HPD intervals: Chen and Shao [33] demonstrated how to use this technique to produce HPD ranges for unknown benefit distribution parameters. To construct time-lapse estimates in this work, samples drawn with the proposed MH method should be employed. For example, a (1 − *γ*%) HPD interval with two points for the 2^th^ parameters of this model can be constructed using the MCMC sampling outputs and the percentile tail points. According to Chen and Shao [33], the BCIs of the parameters of PML distribution *α*, *θ*_1_, *θ*_2_ can be obtained through the following steps:

Step (1): Sorted $\tilde{\alpha }$, $\tilde{\theta_{1}}$, and $\tilde{\theta_{2}}$ as $\left({\tilde{\alpha }}^{\left[1\right]}\leq {\tilde{\alpha }}^{\left[2\right]}\leq \ldots \leq {\tilde{\alpha }}^{\left[A\right]}\right)$, $\left({\tilde{\theta_{1}}}^{\left[1\right]}\leq {\tilde{\theta_{1}}}^{\left[2\right]}\leq \ldots \leq {\tilde{\theta_{1}}}^{\left[A\right]}\right)$ and $\left({\tilde{\theta_{2}}}^{\left[1\right]}\leq {\tilde{\theta_{2}}}^{\left[2\right]}\leq \ldots \leq {\tilde{\theta_{2}}}^{\left[A\right]}\right)$, where *A* denotes the size of the generated of MCMC results
Step (2): The 100(1 − *γ*)% symmetric credible intervals of *α*, *θ*_1_, *θ*_2_ are obtained as $\left({\tilde{\alpha }}^{\left[L\gamma /2\right]},\;{\tilde{\alpha }}^{\left[L\left(1-\gamma /2\right)\right]}\right)$, $\left({\tilde{\theta }}_{1}^{\left[L\gamma /2\right]},\;{\tilde{\theta }}_{1}^{\left[L\left(1-\gamma /2\right)\right]}\right)$ and $\left({\tilde{\theta }}_{2}^{\left[L\gamma /2\right]},\;{\tilde{\theta }}_{2}^{\left[L\left(1-\gamma /2\right)\right]}\right)$

## 7. Simulation

In this part, we simulate to see how each estimate of the vector parameter Ω performs numerically for each method in terms of bias, mean-squared error (MSE), and confidence interval length (L.CI). The following steps are used to create the simulation algorithm of a simple case of PML distribution based on a complete sample.

- The values of the PML distribution parameters Ω=(*α*, *θ*) are as follows:
- Table 1 shows the constant *α*=0.5 and the changes in *θ* to 0.5, 2, and 5.  Table 2 shows the constant *α*=2 and the changes in *θ* to 0.5, 2, and 5.  Table 3 shows the constant *α*=5 and the changes in *θ* to 0.5, 2, and 5.
- The sample size, *n*, is determined. The sample sizes of *n* = 35, 70, and 140 are being considered.
- In LINEX, we consider *c*=−1.5 and 1.5. In entropy, we consider *b*=−1.5 and 1.5.
- The number of replications is determined, that is, *L* = 5000.
- A uniform distribution (*U*) over the interval is used to create random samples of size *n* (0, 1). Then, using the inverse of the distribution function in equation (7), we transform them into samples with a PML distribution with the parameters *α* and *θ*.
- Estimate the parameter of PML distribution; we used the Newton–Raphson algorithm for MLE, and we used MH algorithm in MCMC for Bayesian estimation methods.
- Calculate different measures of performance as bias, MSE, and L.CI for each method.

The following steps are used to create the simulation algorithm of the stress-strength model of PML distribution:

- The values of stress-strength model of PML distribution parameters (*α*, *θ*_1_, *θ*_2_) are as follows:
- Table 4 shows the constant *α*=2 and *θ*_1_=0.75 and the changes in *θ*_2_ to 1.5 and 3.
- Table 5 shows the constant *α*=0.5 and *θ*_1_=2 and the changes in *θ*_2_ to 3 and 5.
- The sample sizes, *n* for strength and *m* for stress, are determined. The sample sizes of (*n*, *m*) = (30, 30), (45, 50), and (70, 60) are being considered.
- In LINEX, we consider *c*=−1.5 and 1.5. In entropy, we consider *b*=−1.5 and 1.5.
- The number of replications is determined, that is, *L* = 5000.
- Generate two uniform distribution (*U*) with interval (0, 1), which is used to create random samples of PML distribution size *n* and *m*. Then, using the inverse of the distribution function in equation (7), we transform them into samples with a PML distribution with the parameters *α* and *θ*_1_ for strength variable and *α* and *θ*_2_ for stress variable.
- Estimate the parameter of PML distribution; we used the Newton–Raphson algorithm for MLE and the Metropolis–Hastings (MH) algorithm in MCMC for Bayesian estimation methods.
- Calculate different measures of performance as mean, MSE, and L.CI for each method.

From the simulation results in Tables 1–5, the conclusions of simulation results are as follows: in all scenarios investigated, the bias, MSE, and L.CI of all estimators drop as sample size increases, indicating an increasing precision in model parameter estimation. In all of the examples studied, Bayesian estimators generated under the assumption of gamma prior are superior to MLE estimators. When compared to Bayesian estimates based on symmetry, asymmetry loss function, and ML estimates, Bayesian estimation based on asymmetry loss function yields more exact results. Also, Bayesian estimates based on the symmetry loss function perform better than the ML estimates. Bayesian estimation under LINEX loss gives best estimators or smaller MSE, minimum L.CI, and minimum bias as compared to the others.

## 8. Applications of Real Data

The derivation of the PML distribution is primarily concerned with its application in data analysis purposes, which makes it useful in a variety of domains, notably those involving lifetime analysis. In this section, we discuss the flexibility of the proposed model for three different applications of real data. This feature is illustrated by taking: firstly, the dataset related to COVID-19 epidemic. Secondly, the analysis of two real datasets of the strength-stress model is described in this section for illustrative purposes.

### 8.1. COVID-19 Data

This is a COVID-19 dataset from the Republic of Moldova that spans 28 days, from October 25 2020 to November 21, 2020. These data formed of the mortality rate of 10000. The data are as follows: 2.0167, 2.2917, 2.1395, 1.4134, 2.6539, 2.4832, 2.5873, 2.5588, 2.0058, 2.4013, 2.6438, 1.6959, 1.9305, 2.0351, 1.1280, 0.2486, 2.3525, 2.2042, 2.4167, 2.2600, 2.1084, 2.1898, 1.4898, 1.8222, 2.1382, 1.9901, 2.0681, and 2.1443.

In this subsection, we compare the fits of the inverse Weibull (IW), Weibull (W), Lomax, PL, generalized Lindley (GL) [34], exponentiated power Lindley (EPL) [35], and PML models in Table 6.  Figure 5 shows the fitted PML, pdf, cdf, and PP plot of these datasets.  Table 7 presents the Bayesian estimation method with different loss functions for parameters of the PML distribution.  Figure 6 shows convergence plots of MCMC for parameter estimates of PML distribution.

By fixing one parameter and adjusting the other, we sketched the log-likelihood for each parameter as shown in Figure 7. The COVID-19 dataset behaves quite well, as the two roots of the parameters are global maximums, as shown in the figures.

### 8.2. Application of Strength-Stress Model

The numerical results of stress-strength reliability estimation for PML distribution for two real datasets are presented in this subsection.

#### 8.2.1. First Data Set

The breaking strengths of jute fibre at two different gauge lengths are shown here. Xia et al. [36] and Saraçoglu et al. [37] employed these two datasets in their study.

The notations used were as follows: breaking strength of jute fibre of gauge length 10 mm can be denoted as *x* “693.73, 704.66, 323.83, 778.17, 123.06, 637.66, 383.43, 151.48, 108.94, 50.16, 671.49, 183.16, 257.44, 727.23, 291.27, 101.15, 376.42, 163.40, 141.38, 700.74, 262.90, 353.24, 422.11, 43.93, 590.48, 212.13, 303.90, 506.60, 530.55, 177.25,” and breaking strength of jute fibre of gauge length 20 mm can be denoted as *y* “71.46, 419.02, 284.64, 585.57, 456.60, 113.85, 187.85, 688.16, 662.66, 45.58, 578.62, 756.70, 594.29, 166.49, 99.72, 707.36, 765.14, 187.13, 145.96, 350.70, 547.44, 116.99, 375.81, 581.60, 119.86, 48.01, 200.16, 36.75, 244.53, 83.55.”

By estimating PML distribution parameters and using the Kolmogorov–Simon test (KST), it was first determined whether or not the PML distribution could be employed to evaluate these datasets. The KST distance values (KSTDV) are small, and the associated *p* values (KSTPV) are larger than 0.05 (see Table 8. Based on the KSTPV, the possibility that the data are from PML distributions cannot be ruled out. Figures 8 and 9 confirm this concluding results of first real data. Figures 10 and 11 confirm that the estimations of *α* and *θ* have global maximum point.

MLE and Bayesian estimation for parameters and reliability value of the strength-stress model of PML distribution are shown in Table 9. We note that the Bayesian estimation methods have the largest reliability value of the strength-stress model of PML distribution and the smallest SE in some loss functions.  Figure 12 shows convergence diagnostics by trace plot and kernel density estimation of the parameters with the normal curve, for 10,000 MCMC iterations.

#### 8.2.2. The Second Data Set

We used real datasets of consumers' waiting times before receiving service from two banks, A and B. Al-Mutairi et al. [28] reported these datasets simultaneously for evaluating the stress-strength reliability in the Lindley distribution. The following are the data: waiting time (in minutes) before customer service in Bank A: *x* is “0.8, 0.8, 1.3, 1.5, 1.8, 1.9, 1.9, 2.1, 2.6, 2.7, 2.9, 3.1, 3.2, 3.3, 3.5, 3.6, 4.0, 4.1, 4.2, 4.2, 4.3, 4.3, 4.4, 4.4, 4.6, 4.7, 4.7, 4.8, 4.9, 4.9, 5.0, 5.3, 5.5, 5.7, 5.7, 6.1, 6.2, 6.2, 6.2, 6.3, 6.7, 6.9, 7.1, 7.1, 7.1, 7.1, 7.4, 7.6, 7.7, 8.0, 8.2, 8.6, 8.6, 8.6, 8.8, 8.8, 8.9, 8.9, 9.5, 9.6, 9.7, 9.8, 10.7, 10.9, 11.0, 11.0, 11.1, 11.2, 11.2, 11.5, 11.9, 12.4, 12.5, 12.9, 13.0, 13.1, 13.3, 13.6, 13.7, 13.9, 14.1, 15.4, 15.4, 17.3, 17.3, 18.1, 18.2, 18.4, 18.9, 19.0, 19.9, 20.6, 21.3, 21.4, 21.9, 23.0, 27.0, 31.6, 33.1, 38.5,” and waiting time (in minutes) before customer service in Bank B: *y* is “0.1, 0.2, 0.3, 0.7, 0.9, 1.1, 1.2, 1.8, 1.9, 2.0, 2.2, 2.3, 2.3, 2.3, 2.5, 2.6, 2.7, 2.7, 2.9, 3.1, 3.1, 3.2, 3.4, 3.4, 3.5, 3.9, 4.0, 4.2, 4.5, 4.7, 5.3, 5.6, 5.6, 6.2, 6.3, 6.6, 6.8, 7.3, 7.5, 7.7, 7.7, 8.0, 8.0, 8.5, 8.5, 8.7, 9.5, 10.7, 10.9, 11.0, 12.1, 12.3, 12.8, 12.9, 13.2, 13.7, 14.5, 16.0, 16.5, 28.0.”

By estimating PML distribution parameters and using the KST, it was first determined whether or not the PML distribution could be employed to evaluate these second datasets. The KSTDV is small, and the associated KSTPV is larger than 0.05 (see Table 10). Based on the KSTPV, the possibility that the data are from PML distributions cannot be ruled out. Figures 13 and 14 confirm this concluding results of the second real data.

Table 11 shows the results of MLE and Bayesian estimation for parameters and the reliability value of the strength-stress model of the PML distribution. In the strength-stress model of the PML distribution, Bayesian estimation approaches have the highest reliability value and the least SE in some loss functions. Convergence diagnostics by trace plot and kernel density estimate of the parameters with the normal curve are shown in Figure 15, for a total of 10,000 MCMC iterations.

## 9. Conclusions

In this article, we introduced a new Lindley distribution that can be abbreviated as PML distribution, and we obtained different properties as moments, moment-generating function, conditional moments, mean deviation, and moments of residual and reversed residual lifetimes. Bayesian and non-Bayesian estimation parameters have been obtained, which the non-Bayesian is a maximum-likelihood estimation. In the case of Bayesian estimation, we perform the approximation using the MCMC technique based on symmetric and asymmetric loss functions. The Bayesian estimator based on gamma priors has been proposed. The confidence intervals have been done for MLE and Bayesian for parameters of model and reliability stress-strength by using the delta method. To test the performance of the different estimators, extensive simulations are run, and it is discovered that all estimators react similarly. In terms of the performance of simulation, Bayesian estimation outperforms MLE in terms of estimating parameters and *R*, according to the simulation study. A comparative study of real datasets shows that PML distribution is well fitted to the considered datasets due to minimum values of KSTDV, CVM, and ADS. Compared with previous studies, we obtained the highest value for *R* compared to previous studies, which indicates the efficiency of the model used and the strength of its interpretation of different data.

In future work, we intend to discuss ranked set sample for PML distribution as Sabry et al. [38], Sabry and Almetwally [39], Hassan et al. [31], Noor-ul-Amin et al. [40], and Esemen et al. [41]. Also, we intend to discuss the inference of PML distribution based on censored sample as Hassan and Ismail [42], Almongy et al. [43] Cho and Lee [44], and Almetwally et al. [45].

## Figures and Tables

**Figure 1:** The pdf and hazard rate with different effects of parameters.

**Figure 2:** LINEX loss function with different values of *c*.

**Figure 3:** Entropy loss function with different values of *b*.

**Figure 4:** Reliability stress-strength model of PML.

**Figure 5:** Estimated pdf and cdf and PP plot for PML distribution for the COVID-19 dataset.

**Figure 6:** MCMC trace and histogram with normal curve of proposed distribution for PML distribution.

**Figure 7:** Existence for the log-likelihood for COVID-19 dataset.

**Figure 8:** Estimated pdf and cdf and PP plot for PML distribution for first data set: strength.

**Figure 9:** Estimated pdf and cdf and PP plot for PML distribution for first dataset: stress.

**Figure 10:** Existence for the log-likelihood for the first dataset: strength.

**Figure 11:** Existence for the log-likelihood for the first dataset: stress.

**Figure 12:** MCMC trace and histogram with normal curve of proposed distribution for PML distribution for the first dataset.

**Figure 13:** Estimated pdf and cdf and PP plot for PML distribution for the second dataset: strength.

**Figure 14:** Estimated pdf and cdf and PP plot for PML distribution for the second dataset: stress.

**Figure 15:** MCMC trace and Histogram with normal curve of proposed distribution for PML distribution for the second dataset.

**Table 1:** Bayesian with different loss functions and MLE of the parameters of PML distribution when *α*=0.5.

*α*=0.5			MLE			SE			LINEX *c* = −1.5			LINEX *c* = 1.5			Entropy *b* = 1.5			Entropy *b* = −1.5		
*θ*			Bias	MSE	L.CI	Bias	MSE	L.CI	Bias	MSE	L.CI	Bias	MSE	L.CI	Bias	MSE	L.CI	Bias	MSE	L.CI
0.5	35	*α*	0.0385	0.0067	0.2834	−0.0138	0.0012	0.1193	−0.0118	0.0012	0.1210	−0.0158	0.0013	0.1172	−0.0125	0.0012	0.1200	−0.0207	0.0014	0.1149
		*θ*	−0.1404	0.0232	0.2322	−0.0552	0.0036	0.0921	−0.0526	0.0034	0.0940	−0.0578	0.0039	0.0913	−0.0533	0.0034	0.0929	−0.0648	0.0047	0.0893
	70	*α*	0.0281	0.0029	0.1811	−0.0168	0.0008	0.0802	−0.0158	0.0007	0.0807	−0.0177	0.0008	0.0801	−0.0161	0.0007	0.0805	−0.0200	0.0009	0.0798
		*θ*	−0.1395	0.0213	0.1674	−0.0572	0.0035	0.0758	−0.0559	0.0032	0.0761	−0.0585	0.0038	0.0754	−0.0563	0.0033	0.0758	−0.0620	0.0042	0.0750
	140	*α*	0.0214	0.0015	0.1287	0.0020	0.0003	0.0638	0.0026	0.0003	0.0645	0.0014	0.0003	0.0633	0.0024	0.0003	0.0641	−0.0001	0.0003	0.0624
		*θ*	−0.1379	0.0199	0.1170	−0.1097	0.0126	0.0876	−0.1085	0.0123	0.0876	−0.1109	0.0013	0.0706	−0.1086	0.0012	0.0705	−0.1147	0.0014	0.0689

2	35	*α*	0.0637	0.0146	0.4028	0.0547	0.0072	0.2352	0.0587	0.0079	0.2408	0.0507	0.0066	0.2300	0.0570	0.0076	0.2374	0.0429	0.0057	0.2247
		*θ*	−0.7108	0.5422	0.7543	−0.3937	0.1978	0.7775	−0.3500	0.1615	0.7368	−0.4348	0.2353	0.8184	−0.3845	0.1895	0.7663	−0.4391	0.2414	0.8437
	70	*α*	0.0582	0.0083	0.2742	0.0520	0.0047	0.1736	0.0537	0.0050	0.1754	0.0502	0.0045	0.1714	0.0530	0.0049	0.1743	0.0466	0.0041	0.1699
		*θ*	−0.5727	0.4577	0.5249	−0.2578	0.0863	0.5356	−0.2375	0.0737	0.4948	−0.2774	0.0993	0.5708	−0.2538	0.0836	0.5245	−0.2776	0.0998	0.5795
	140	*α*	0.0452	0.0044	0.1897	0.0428	0.0027	0.1159	0.0437	0.0028	0.1167	0.0419	0.0027	0.1150	0.0434	0.0028	0.1160	0.0401	0.0025	0.1138
		*θ*	−0.4298	0.3560	0.3538	−0.2930	0.0853	0.3661	−0.2726	0.0782	0.3351	−0.3125	0.0853	0.3981	−0.2890	0.0793	0.3592	−0.3127	0.0884	0.4025

5	35	*α*	0.0267	0.0139	0.4498	0.1260	0.0210	0.2666	0.1289	0.0218	0.2678	0.1231	0.0201	0.2640	0.1275	0.0214	0.2667	0.1184	0.0188	0.2609
		*θ*	−2.1849	1.3128	2.8811	−0.1970	0.1548	1.3190	−0.1455	0.1282	1.2454	−0.2484	0.1891	1.3406	−0.1932	0.1524	1.3090	−0.2158	0.1678	1.3355
	70	*α*	0.0180	0.0071	0.3240	0.1195	0.0163	0.1765	0.1211	0.0167	0.1801	0.1180	0.0159	0.1747	0.1204	0.0165	0.1776	0.1152	0.0152	0.1730
		*θ*	−2.2569	0.6368	2.0546	−0.0928	0.0364	0.6300	−0.0803	0.0323	0.6044	−0.1054	0.0408	0.6510	−0.0920	0.0361	0.6263	−0.0972	0.0379	0.6426
	140	*α*	0.0123	0.0038	0.2362	0.1183	0.0151	0.1261	0.1192	0.0154	0.1272	0.1174	0.0149	0.1248	0.1188	0.0152	0.1266	0.1158	0.0145	0.1227
		*θ*	−2.3325	0.4565	1.3810	−0.1221	0.0309	0.4782	−0.1123	0.0274	0.4541	−0.1320	0.0347	0.5026	−0.1214	0.0307	0.4765	−0.1255	0.0322	0.4863

**Table 2:** Bayesian with different loss functions and MLE of the parameters of PML distribution when *α*=2.

*α*=2			MLE			SE			LINEX *c* = −1.5			LINEX *c* = 1.5			Entropy *b* = 1.5			Entropy *b* = −1.5		
*α*			Bias	MSE	L.CI	Bias	MSE	L.CI	Bias	MSE	L.CI	Bias	MSE	L.CI	Bias	MSE	L.CI	Bias	MSE	L.CI
0.5	35	*α*	0.1588	0.0958	1.0420	0.0167	0.0262	0.6064	0.0372	0.0287	0.6197	−0.0038	0.0249	0.5905	0.0200	0.0265	0.6048	−0.0004	0.0255	0.5970
		*θ*	−0.1411	0.0232	0.2259	−0.1019	0.0131	0.1964	−0.0981	0.0124	0.1991	−0.1055	0.0137	0.1944	−0.0988	0.0125	0.1968	−0.1170	0.0163	0.1944
	70	*α*	0.1136	0.0470	0.7247	−0.0078	0.0112	0.4110	−0.0012	0.0114	0.4180	−0.0143	0.0112	0.4060	−0.0067	0.0112	0.4117	−0.0132	0.0113	0.4100
		*θ*	−0.1392	0.0210	0.1578	−0.1014	0.0115	0.1352	−0.0996	0.0111	0.1348	−0.1031	0.0118	0.1347	−0.0999	0.0112	0.1345	−0.1087	0.0130	0.1361
	140	*α*	0.0848	0.0232	0.4955	−0.0059	0.0059	0.2925	−0.0022	0.0059	0.2938	−0.0097	0.0059	0.2920	−0.0053	0.0059	0.2925	−0.0091	0.0059	0.2935
		*θ*	−0.1374	0.0198	0.1168	−0.1058	0.0102	0.0987	−0.1048	0.0102	0.0984	−0.1069	0.0102	0.0984	−0.1049	0.0102	0.0984	−0.1102	0.0113	0.1003

2	35	*α*	0.3502	0.2374	1.3285	0.1448	0.0623	0.7860	0.1735	0.0758	0.8153	0.1158	0.0510	0.7319	0.1492	0.0641	0.7901	0.1223	0.0544	0.7577
		*θ*	−0.6781	0.5048	0.8315	−0.4012	0.2009	0.7545	−0.3579	0.1644	0.7206	−0.4415	0.2381	0.7845	−0.3921	0.1927	0.7455	−0.4458	0.2440	0.8015
	70	*α*	0.2953	0.1419	0.9176	0.0908	0.0242	0.4890	0.0998	0.0268	0.5008	0.0817	0.0217	0.4790	0.0922	0.0245	0.4904	0.0836	0.0223	0.4829
		*θ*	−0.7166	0.3132	0.5237	−0.2672	0.0887	0.5129	−0.2452	0.0750	0.4751	−0.2885	0.1031	0.5477	−0.2628	0.0858	0.5048	−0.2888	0.1037	0.5550
	140	*α*	0.2630	0.0959	0.6414	0.0925	0.0171	0.3505	0.0982	0.0187	0.3542	0.0868	0.0156	0.3417	0.0934	0.0173	0.3504	0.0880	0.0160	0.3456
		*θ*	−0.7314	0.2544	0.3688	−0.3050	0.0810	0.3775	−0.2833	0.0688	0.3502	−0.3256	0.0912	0.4059	−0.3007	0.0800	0.3715	−0.3259	0.0912	0.4099

5	35	*α*	0.3374	0.2188	1.2717	0.4257	0.2162	0.6873	0.4670	0.2610	0.7408	0.3818	0.1735	0.6232	0.4315	0.2221	0.6929	0.3956	0.1871	0.6459
		*θ*	−0.8913	1.0727	2.7626	−0.2557	0.1920	1.3448	−0.1972	0.1483	1.2275	−0.3136	0.2443	1.4873	−0.2514	0.1880	1.3381	−0.2777	0.2125	1.4168
	70	*α*	0.2888	0.1389	0.9240	0.2880	0.0952	0.4242	0.3066	0.1082	0.4515	0.2685	0.0825	0.3920	0.2907	0.0971	0.4275	0.2739	0.0861	0.4046
		*θ*	−0.6005	0.8241	1.8491	−0.1265	0.0412	0.5910	−0.1135	0.0356	0.5534	−0.1395	0.0474	0.6262	−0.1256	0.0408	0.5888	−0.1311	0.0434	0.6012
	140	*α*	0.2794	0.1009	0.5928	0.3125	0.1050	0.3305	0.3295	0.1172	0.3578	0.2943	0.0927	0.3033	0.3150	0.1068	0.3341	0.2994	0.0961	0.3108
		*θ*	−0.2022	0.4182	1.2060	−0.1524	0.0403	0.4920	−0.1408	0.0352	0.4578	−0.1640	0.0457	0.5172	−0.1516	0.0399	0.4907	−0.1565	0.0422	0.5045

**Table 3:** Bayesian with different loss functions and MLE of the parameters of PML distribution when *α*=5.

*α*=5			MLE			SE			LINEX *c* = −1.5			LINEX *c* = 1.5			Entropy *b* = 1.5			Entropy *b* = −1.5		
*θ*			Bias	MSE	L.CI	Bias	MSE	L.CI	Bias	MSE	L.CI	Bias	MSE	L.CI	Bias	MSE	L.CI	Bias	MSE	L.CI
0.5	35	*α*	0.4024	0.6295	2.6819	−0.0660	0.0885	1.1394	−0.0312	0.0838	1.0916	−0.1009	0.0957	1.1372	−0.0636	0.0879	1.1390	−0.0781	0.0913	1.1494
		*θ*	−0.1433	0.0241	0.2332	−0.0605	0.0045	0.1144	−0.0654	0.0045	0.1160	−0.0627	0.0048	0.1135	−0.0888	0.0049	0.1154	−0.0688	0.0056	0.1123
	70	*α*	0.2854	0.2961	1.8169	−0.0360	0.0234	0.5831	−0.0266	0.0225	0.5750	−0.0454	0.0246	0.5889	−0.0354	0.0233	0.5830	−0.0392	0.0238	0.5878
		*θ*	−0.1402	0.0214	0.1631	−0.0641	0.0046	0.0848	−0.0630	0.0045	0.0855	−0.0652	0.0047	0.0840	−0.0633	0.0045	0.0853	−0.0682	0.0051	0.0838
	140	*α*	0.2293	0.1601	1.2861	−0.0412	0.0154	0.4555	−0.0353	0.0147	0.4469	−0.0471	0.0163	0.4586	−0.0408	0.0154	0.4552	−0.0432	0.0157	0.4568
		*θ*	−0.1385	0.0201	0.1183	−0.0660	0.0045	0.0603	−0.0583	0.0043	0.0604	−0.0665	0.0047	0.0604	−0.0655	0.0041	0.0603	−0.0681	0.0049	0.0603

2	35	*α*	0.8560	1.4906	3.4142	0.0982	0.1093	1.2442	0.1412	0.1273	1.3106	0.0552	0.0967	1.1502	0.1011	0.1102	1.2461	0.0840	0.1054	1.2200
		*θ*	−0.6798	0.5093	0.8516	−0.2332	0.0662	0.4068	−0.2132	0.0572	0.4055	−0.2530	0.0761	0.4227	−0.2294	0.0644	0.4066	−0.2523	0.0760	0.4277
	70	*α*	0.7575	0.9454	2.3907	0.0330	0.0199	0.5286	0.0405	0.0209	0.5308	0.0254	0.0190	0.5178	0.0335	0.0199	0.5293	0.0305	0.0196	0.5234
		*θ*	−0.3717	0.3316	0.5429	−0.1602	0.0324	0.3165	−0.1518	0.0294	0.3060	−0.1685	0.0354	0.3240	−0.1587	0.0318	0.3139	−0.1678	0.0352	0.3243
	140	*α*	0.6567	0.5930	1.5770	0.0198	0.0060	0.3259	0.0221	0.0063	0.3328	0.0175	0.0057	0.3196	0.0200	0.0060	0.3260	0.0191	0.0059	0.3247
		*θ*	−0.2831	0.2427	0.3610	−0.0836	0.0154	0.2443	−0.0802	0.0142	0.2348	−0.0869	0.0166	0.2524	−0.0830	0.0152	0.2425	−0.0866	0.0166	0.2520

5	35	*α*	0.8108	1.3241	3.2024	0.3466	0.2031	1.1142	0.4058	0.2674	1.2388	0.2862	0.1482	0.9942	0.3503	0.2068	1.1177	0.3278	0.1854	1.0741
		*θ*	−0.8697	1.5047	2.9120	−0.2885	0.1730	1.1422	−0.2337	0.1309	1.0563	−0.3428	0.2226	1.2414	−0.2845	0.1694	1.1366	−0.3090	0.1918	1.1956
	70	*α*	0.7320	0.8286	2.1220	0.1328	0.0368	0.5350	0.1440	0.0418	0.5542	0.1216	0.0321	0.5113	0.1335	0.0371	0.5359	0.1292	0.0353	0.5292
		*θ*	−0.5986	0.8153	1.8003	−0.1232	0.0332	0.5215	−0.1127	0.0293	0.4989	−0.1337	0.0375	0.5388	−0.1225	0.0329	0.5202	−0.1269	0.0347	0.5284
	140	*α*	0.6731	0.6083	1.5453	0.1335	0.0278	0.3640	0.1409	0.0308	0.3841	0.1259	0.0249	0.3514	0.1339	0.0280	0.3652	0.1310	0.0268	0.3601
		*θ*	−0.4410	0.6281	1.2586	−0.1139	0.0238	0.3918	−0.1069	0.0212	0.3770	−0.1209	0.0265	0.4080	−0.1134	0.0236	0.3904	−0.1164	0.0247	0.3969

**Table 4:** Bayesian with different loss functions and MLE of the parameters of strength-stress model of PML distribution when *α*=2, *θ*_1_=0.75.

*α*=2, *θ*_1_=0.75			MLE			SE			LINEX *c* = −1.5			LINEX *c* = 1.5			Entropy *b* = 1.5			Entropy *b* = −1.5		
*θ*_2_	*n*, *m*		Mean	MSE	L.CI	Mean	MSE	L.CI	Mean	MSE	L.CI	Mean	MSE	L.CI	Mean	MSE	L.CI	Mean	MSE	L.CI
1.5	30, 30	*α*	2.1767	0.0725	0.7981	1.7675	0.0763	0.5754	1.7906	0.0667	0.5810	1.7447	0.0869	0.5680	1.7719	0.0743	0.5741	1.7455	0.0870	0.5758
		*θ*_1_	0.5268	0.0578	0.3509	0.6514	0.0131	0.2055	0.6586	0.0119	0.2103	0.6444	0.0144	0.2025	0.6550	0.0124	0.2066	0.6333	0.0168	0.2037
		*θ*_2_	0.5171	0.9728	0.3203	1.0580	0.1967	0.1371	1.0715	0.1851	0.1385	1.0458	0.2076	0.1360	1.0620	0.1932	0.1365	1.0391	0.2137	0.1386
		*R*	0.4820	0.0355	0.2808	0.6101	0.0032	0.1190	0.6097	0.0033	0.1209	0.6108	0.0031	0.1171	0.6092	0.0033	0.1186	0.6154	0.0027	0.1147
	45, 50	*α*	2.1766	0.0631	0.7016	1.8279	0.0450	0.4761	1.8378	0.0408	0.4666	1.8181	0.0492	0.4817	1.8297	0.0441	0.4725	1.8187	0.0491	0.4858
		*θ*_1_	0.5170	0.0584	0.2536	0.6467	0.0133	0.1897	0.6508	0.0124	0.1908	0.6426	0.0141	0.1886	0.6488	0.0128	0.1897	0.6360	0.0156	0.1897
		*θ*_2_	0.5206	0.9623	0.2189	1.1273	0.1426	0.2033	1.1445	0.1299	0.1879	1.1121	0.1543	0.1902	1.1320	0.1390	0.1912	1.1055	0.1595	0.1892
			0.4907	0.0304	0.2144	0.6302	0.0017	0.1190	0.6322	0.0016	0.1221	0.6287	0.0018	0.1164	0.6302	0.0017	0.1205	0.6308	0.0017	0.1210
	70, 60	*α*	2.1471	0.0429	0.5727	1.8341	0.0382	0.4187	1.8416	0.0351	0.4077	1.8269	0.0413	0.4232	1.8355	0.0376	0.4174	1.8274	0.0411	0.4240
		*θ*_1_	0.5148	0.0578	0.1978	0.6471	0.0122	0.1496	0.6499	0.0116	0.1493	0.6443	0.0128	0.1513	0.6485	0.0119	0.1487	0.6400	0.0137	0.1514
		*θ*_2_	0.5216	0.9607	0.2128	1.1528	0.1230	0.1971	1.1696	0.1115	0.1902	1.1378	0.1338	0.2027	1.1574	0.1198	0.1980	1.1317	0.1384	0.2058
		*R*	0.4917	0.0291	0.1772	0.6362	0.0010	0.0975	0.6387	0.0009	0.0938	0.6341	0.0011	0.1001	0.6365	0.0010	0.0958	0.6350	0.0011	0.1020

3	30, 30	*α*	2.1926	0.0765	0.7804	1.5812	0.2452	0.7572	1.6011	0.2242	0.7295	1.5637	0.2642	0.7795	1.5854	0.2406	0.7506	1.5612	0.2676	0.7855
		*θ*_1_	0.5237	0.0623	0.4136	0.6995	0.0075	0.1797	0.7056	0.0070	0.1824	0.6935	0.0080	0.1780	0.7024	0.0072	0.1797	0.6849	0.0093	0.1783
		*θ*_2_	0.5175	6.1763	0.4578	2.4610	0.3802	0.3813	2.4879	0.3439	0.3683	2.4396	0.4101	0.3839	2.4643	0.3755	0.3806	2.4453	0.4022	0.3829
		*R*	0.4834	0.1143	0.2717	0.7931	0.0010	0.0695	0.7932	0.0010	0.0715	0.7935	0.0010	0.0682	0.7923	0.0010	0.0704	0.7973	0.0008	0.0669
	45, 50	*α*	2.1749	0.0537	0.5967	1.7872	0.0939	0.5623	1.8002	0.0826	0.5318	1.7757	0.1044	0.5936	1.7899	0.0915	0.5545	1.7749	0.1053	0.5984
		*θ*_1_	0.5164	0.0582	0.2372	0.7062	0.0055	0.1866	0.7085	0.0051	0.1851	0.7038	0.0059	0.1880	0.7073	0.0053	0.1852	0.7002	0.0066	0.1934
		*θ*_2_	0.5152	1.1776	0.2244	2.6988	0.1795	0.2071	2.7290	0.1451	0.1963	2.6729	0.2117	0.2078	2.7027	0.1748	0.2070	2.6803	0.2024	0.2076
		*R*	0.5878	0.1096	0.2108	0.8086	0.0003	0.0760	0.8101	0.0003	0.0718	0.8074	0.0004	0.0799	0.8085	0.0003	0.0749	0.8093	0.0003	0.0797
	70, 60	*α*	2.1722	0.0529	0.5996	1.7880	0.0856	0.5212	1.8008	0.0753	0.4840	1.7764	0.0953	0.5573	1.7906	0.0835	0.5118	1.7759	0.0959	0.5609
		*θ*_1_	0.5208	0.0552	0.2035	0.6991	0.0060	0.1729	0.7012	0.0056	0.1713	0.6971	0.0063	0.1721	0.7001	0.0058	0.1723	0.6939	0.0070	0.1717
		*θ*_2_	0.5170	0.5168	0.2249	2.6922	0.1715	0.2068	2.7246	0.1372	0.1861	2.6630	0.2054	0.2074	2.6964	0.1667	0.1967	2.6717	0.1951	0.1972
		*R*	0.6849	0.1011	0.1896	0.8108	0.0002	0.0594	0.8125	0.0002	0.0590	0.8093	0.0003	0.0620	0.8108	0.0002	0.0596	0.8112	0.0002	0.0626

**Table 5:** Bayesian with different loss functions and MLE of the parameters of strength-stress model of PML distribution when *α*=0.5, *θ*_1_=2.

*α*=0.5, *θ*_1_=2			MLE			SE			LINEX *c* = −1.5			LINEX *c* = 1.5			Entropy *b* = 1.5			Entropy *b* = −1.5		
*θ*_2_	*n*, *m*		Mean	MSE	L.CI	Mean	MSE	L.CI	Mean	MSE	L.CI	Mean	MSE	L.CI	Mean	MSE	L.CI	Mean	MSE	L.CI
3	30, 30	*α*	0.5566	0.0274	0.3420	0.5833	0.0125	0.2735	0.5866	0.0132	0.2777	0.5800	0.0128	0.2693	0.5852	0.0128	0.2749	0.5740	0.0108	0.2663
		*θ*_1_	1.2718	0.5734	0.8148	1.6300	0.1645	0.5845	1.6701	0.1368	0.5859	1.5916	0.1940	0.5707	1.6381	0.1584	0.5796	1.5894	0.1970	0.5786
		*θ*_2_	1.3005	2.9300	0.7999	2.2860	0.5355	0.5929	2.3692	0.4232	0.5906	2.2171	0.6395	0.5939	2.2972	0.5194	0.5872	2.2335	0.6148	0.5999
		*R*	0.4017	0.0131	0.3148	0.4798	0.0023	0.1719	0.4813	0.0022	0.1702	0.4797	0.0024	0.1752	0.4793	0.0022	0.1703	0.4828	0.0024	0.1780
	45, 50	*α*	0.5548	0.0266	0.2354	0.5959	0.0124	0.2119	0.5979	0.0132	0.2165	0.5938	0.0122	0.2075	0.5970	0.0129	0.2139	0.5901	0.0107	0.2037
		*θ*_1_	1.2808	0.5465	0.6710	1.8178	0.0591	0.6087	1.8337	0.0513	0.5859	1.8022	0.0672	0.6426	1.8208	0.0574	0.6020	1.8027	0.0674	0.6465
		*θ*_2_	1.2766	2.9925	0.5888	2.6919	0.1212	0.5631	2.7222	0.0985	0.5468	2.6624	0.1455	0.5682	2.6958	0.1180	0.6225	2.6726	0.1374	0.6068
		*R*	0.3927	0.0124	0.2543	0.4878	0.0020	0.1664	0.4879	0.0017	0.1578	0.4877	0.0022	0.1791	0.4875	0.0019	0.1645	0.4889	0.0022	0.1784
	70, 60	*α*	0.5538	0.0254	0.1965	0.5987	0.0123	0.1910	0.6004	0.0126	0.1992	0.5971	0.0119	0.1980	0.5996	0.0125	0.2004	0.5941	0.0105	0.1934
		*θ*_1_	1.2713	0.5472	0.4981	1.8257	0.0442	0.4410	1.8375	0.0388	0.4195	1.8139	0.0498	0.4652	1.8279	0.0431	0.4380	1.8145	0.0497	0.4676
		*θ*_2_	1.2728	3.0028	0.5513	2.7485	0.0824	0.5400	2.7694	0.0690	0.4990	2.7281	0.0965	0.5783	2.7512	0.0806	0.5347	2.7355	0.0915	0.5658
		*R*	0.3938	0.0112	0.2200	0.4926	0.0011	0.1251	0.4925	0.0010	0.1170	0.4928	0.0013	0.1332	0.4924	0.0011	0.1244	0.4937	0.0013	0.1329

5	30, 30	*α*	0.5610	0.0310	0.3112	0.6233	0.0228	0.3032	0.6264	0.0238	0.2934	0.6201	0.0218	0.3027	0.6249	0.0233	0.3134	0.6150	0.0204	0.3112
		*θ*_1_	1.2998	0.5308	0.7903	1.6605	0.1533	0.6998	1.6998	0.1286	0.7047	1.6227	0.1801	0.7010	1.6684	0.1479	0.7022	1.6211	0.1828	0.7146
		*θ*_2_	1.2868	1.8219	0.8729	3.9871	1.0962	0.7302	4.1680	0.7444	0.7852	3.8498	1.4090	0.7903	4.0009	1.0668	0.9612	3.9223	1.2401	0.9501
		*R*	0.3891	0.0715	0.3059	0.6464	0.0017	0.1597	0.6509	0.0016	0.1509	0.6445	0.0018	0.1656	0.6457	0.0016	0.1576	0.6502	0.0018	0.1672
	45, 50	*α*	0.5578	0.0271	0.2952	0.6135	0.0224	0.2955	0.6373	0.0225	0.2899	0.6329	0.0213	0.2928	0.6362	0.0224	0.2970	0.6292	0.0202	0.2880
		*θ*_1_	1.2701	0.5566	0.6059	1.8277	0.0473	0.5174	1.8431	0.0403	0.4866	1.8126	0.0548	0.5371	1.8306	0.0459	0.5133	1.8131	0.0548	0.5404
		*θ*_2_	1.2869	1.0809	0.7585	4.6279	0.1690	0.6344	4.6712	0.1318	0.5441	4.5852	0.2103	0.7264	4.6311	0.1661	0.6272	4.6118	0.1842	0.6756
		*R*	0.3984	0.0643	0.2328	0.6545	0.0008	0.1008	0.6542	0.0007	0.0952	0.6547	0.0009	0.1067	0.6541	0.0008	0.1001	0.6563	0.0010	0.1064
	70, 60	*α*	0.5532	0.0259	0.2770	0.6267	0.0207	0.2534	0.6285	0.0213	0.2582	0.6249	0.0201	0.2482	0.6276	0.0210	0.2556	0.6217	0.0191	0.2410
		*θ*_1_	1.2862	0.5268	0.5165	1.8445	0.0382	0.4573	1.8561	0.0334	0.4354	1.8329	0.0434	0.4786	1.8467	0.0372	0.4538	1.8335	0.0433	0.4795
		*θ*_2_	1.2716	0.9182	0.5106	4.6996	0.1070	0.4726	4.7290	0.0868	0.4374	4.6701	0.1295	0.5243	4.7017	0.1054	0.4701	4.6888	0.1150	0.4898
		*R*	0.3887	0.0681	0.1938	0.6556	0.0007	0.0942	0.6552	0.0006	0.0900	0.6560	0.0008	0.0981	0.6554	0.0007	0.0936	0.6571	0.0008	0.0978

**Table 6:** MLE, CvMS, ADS, and KST for different alternative models of PML distribution.

		Estimates	SE	KSTDV	KSTPV	CVMS	ADS
PML	*α*	3.7674	0.5197	**0.1332**	**0.6545**	**0.2066**	**1.2336**
	*θ*	0.0562	0.0246				

IW	*β*	1.3247	0.1494	0.3645	0.0008	1.0667	5.6951
	*λ*	1.6520	0.3131				

W	*β*	5.2397	0.8497	0.1877	0.2446	0.2858	1.4193
	*λ*	2.2112	0.0821				

Lomax	*β*	18597045.81	36.1753	0.4266	0.0000	0.4855	2.7928
	*λ*	38134939.97	10.5566				

PL	*β*	3.8650	0.5334	0.1723	0.3375	0.2642	1.3997
	*θ*	0.0947	0.0421				

GL	*γ*	6.7549	2.2383	0.2644	0.0323	0.5405	3.0780
	*λ*	1.5801	0.1978				

EPL	*α*	0.21173	0.05778	0.1534	0.4783	0.2726	1.3950
	*θ*	0.00018	0.00049				
	*β*	9.98403	0.02596				

**Table 7:** Bayesian for parameters of PML distribution with different loss functions.

	SELF		LINEC *c* = −1.5		LINEC *c* = 1.5		Entropy *b* = −1.5		Entropy *b* = 1.5	
	Estimates	SE	Estimates	SE	Estimates	SE	Estimates	SE	Estimates	SE
*α*	3.7586	0.4156	3.8948	0.4921	3.6364	0.0022	3.7700	0.4877	3.7016	0.4194
*θ*	0.0592	0.0194	0.0594	0.0262	0.0589	0.0216	0.0607	0.0352	0.0509	0.0171

**Table 8:** MLE with SE and KST with *p* value for the first data.

	*X*				*Y*			
	Estimates	SE	KSTDV	KSTPV	Estimates	SE	KSTDV	KSTPV
*α*	1.0274	0.0328	0.1188	0.7470	0.8626	0.0792	0.1325	0.6204
*θ*	0.0025	0.0004			0.0073	0.0035		

**Table 9:** MLE and Bayesian for parameter and reliability of the strength-stress model of PML distribution: first dataset.

	MLE		SELF		LINEC *c* = −1.5		LINEC *c* = 1.5		Entropy *c* = −1.5		Entropy *c* = 1.5	
	Estimates	SE	Estimates	SE	Estimates	SE	Estimates	SE	Estimates	SE	Estimates	SE
*α*	0.9353	0.0412	0.9273	0.0407	0.9290	0.2363	0.9257	0.0143	0.9279	0.0973	0.9244	5.1811
*θ*_1_	0.0044	0.0011	0.0048	0.0010	0.0048	0.0018	0.0048	0.0011	0.0049	0.0013	0.0042	0.0062
*θ*_2_	0.0047	0.0012	0.0052	0.0011	0.0052	0.0020	0.0052	0.0020	0.0053	0.5020	0.0045	0.0061
*R*	0.6284		0.6303		0.6303		0.6303		0.6309		0.6260	

**Table 10:** MLE with SE and KST with *p* value for the first data.

	*X*				*Y*			
	Estimates	SE	KSS	*p* value KS	Estimates	SE	KSS	*p* value KS
*α*	1.0525	0.0681	0.1216	0.1041	0.9461	0.0812	0.1431	0.1709
*θ*	0.0904	0.0163			0.1715	0.0315		

**Table 11:** MLE and Bayesian for parameter and reliability of strength-stress model of PML distribution: the second dataset.

	MLE		SELF		LINEC *c* = −1.5		LINEC *c* = 1.5		Entropy *c* = −1.5		Entropy *c* = 1.5	
	Estimates	SE	Estimates	SE	Estimates	SE	Estimates	SE	Estimates	SE	Estimates	SE
*α*	1.0102	0.0522	1.0066	0.0541	1.0088	0.3028	1.0044	0.0147	1.0073	5.3167	1.0030	5.3488
*θ*_1_	0.1002	0.0144	0.1023	0.0166	0.1025	0.0239	0.1021	0.0174	0.1030	24.8112	0.0990	0.2491
*θ*_2_	0.1510	0.0209	0.1543	0.0264	0.1548	0.0413	0.1538	0.0253	0.1554	15.8021	0.1489	0.3689
*R*	0.6940		0.6937		0.6940		0.6934		0.6937		0.6940	

## Data Availability

The data used to support the findings of this study are included in the article.
